The article "COVID-19 Epidemic in Sri Lanka: A Mathematical and Computational Modelling Approach to Control" was published in 2020. Journal: Comput Math Methods Med.

# COVID-19 Epidemic in Sri Lanka: A Mathematical and Computational Modelling Approach to Control

**DOI:** 10.1155/2020/4045064

**Published:** 2020-10-16

**Authors:** W. P. T. M. Wickramaarachchi, S. S. N. Perera, S. Jayasinghe

**Affiliations:** ^1^Department of Mathematics, The Open University of Sri Lanka, Nawala, Nugegoda, Sri Lanka; ^2^Department of Mathematics, University of Colombo, Colombo 03, Sri Lanka; ^3^Department of Clinical Medicine, University of Colombo, Colombo 03, Sri Lanka

## Abstract

The ongoing COVID-19 outbreak that originated in the city of Wuhan, China, has caused a significant damage to the world population and the global economy. It has claimed more than 0.8 million lives worldwide, and more than 27 million people have been infected as of 07^th^ September 2020. In Sri Lanka, the first case of COVID-19 was reported late January 2020 which was a Chinese national and the first local case was identified in the second week of March. Since then, the government of Sri Lanka introduced various sequential measures to improve social distancing such as closure of schools and education institutes, introducing work from home model to reduce the public gathering, introducing travel bans to international arrivals, and more drastically, imposed island wide curfew expecting to minimize the burden of the disease to the Sri Lankan health system and the entire community. Currently, there are 3123 cases with 12 fatalities and also, it was reported that 2925 patients have recovered and are discharged from hospitals, according to the Ministry of Health, Sri Lanka. In this study, we use the SEIR conceptual model and its modified version by decomposing infected patients into two classes: patients who show mild symptoms and patients who tend to face severe respiratory problems and are required to be treated in intensive care units. We numerically simulate the models for about a five-month period reflecting the early stage of the epidemic in the country, considering three critical parameters of COVID-19 transmission mainly in the Sri Lankan context: efficacy of control measures, rate of overseas imported cases, and time to introduce social distancing measures by the respective authorities.

## 1. Introduction

Sri Lanka periodically faces epidemics of infections that cause morbidity and mortality. There is epidemiological data on specific diseases such as leptospirosis and dengue. Though clinicians observe periodic epidemics of influenza and other respiratory illnesses, there is scarce information on their spread and case fatality rates or numbers. This is partly because respiratory illnesses are quite common and regular diagnostic tests are rarely available in the state sector hospitals. Nevertheless, Sri Lanka seems to have escaped major viral epidemic respiratory illnesses such as severe acute respiratory syndrome (SARS) and Middle East respiratory syndrome (MERS) until COVID-19 was detected in a Sri Lankan tour guide on the 10^th^ of March 2020. However, the country had not been impacted by SARS and MERS significantly that emerged two decades ago since those outbreaks were contained and they had not spread across the world to become a global pandemic [1, 2].

Since the SARS epidemic outbreak of SARS, 18 years ago, a large number of similar viruses have been discovered in bats, in which its natural reservoir host is bats [3]. A new coronavirus disease 2019 (COVID-19) is caused by severe acute respiratory syndrome coronavirus 2 (SARS-COV-2), and research and investigations lead by the WHO are still ongoing to identify the origin of the novel coronavirus. Given the significant sequence similarity between the SARS-CoV-2 and the SARS-like bat coronavirus from *Hipposideros* bats found in China, the natural host of the SARS-CoV-2 pathogen was assumed to be the *Hipposideros* bat [4].

The virus spreads from human-to-human via droplets or through contaminated surfaces which in turn enter the nasal mucosa, oral cavity, or mucosa of the eyes through touch. This is similar to the spread of influenza (e.g., H1N1) and SARS. However, the COVID-19 potential of transmission is much higher since it is found to be very contagious [5]. As a result, the estimated doubling times range from 6.4 to 7.4 days [6].

The disease is characterized by cough, fever, and sore throat and may result in virus-induced pneumonia and progressive respiratory failure owing to alveolar damage caused by the virus. As a result, the mortality rates from the illness are also relatively high. The disease is also characterized by a mean incubation period of 5.2 days (95% confidence interval (CI), 4.1 to 7.0) [7].

The proportion of asymptomatic cases reached 30.8% (confidence interval 7.7% to 53.8%) [8]. It is found that the virus is shed throughout the illness. As a result, the virus is more infective for a longer duration than other illnesses. Milder cases cleared the virus by 10 days while 90% of severe cases continued to shed the virus in the nasal secretions beyond 10 days from the onset of illness [9–11].

Briefing the COVID-19 situation in Sri Lanka, the index case was a Chinese tourist who was detected with the illness on the 27^th^ of January and admitted to the National Infection Disease Hospital. The first Sri Lankan patient known to be a tourist guide who had not traveled overseas was detected to have the illness on the 11^th^ of March. Having understood the potential spread of the disease over the entire population is Sri Lanka, the government of Sri Lanka took immediate sequential measures such as island-wide school closure, travel ban from selected countries (South Korea, Italy, and Iran), declaration of special holidays to limit public gathering, shutting down the Colombo International Airport for all arrivals to the island, and finally deciding to impose island-wide curfew. As of 07^th^ September 2020, there are 3123 confirmed cases of COVID-19, 12 deaths, and 2975 recoveries [12].

Since Sri Lanka has been a developing country, the facilities to treat COVID-19 patients are found to be very limited. Therefore, it is very critical to understand how sequential control measures should be introduced and in which capacity and efficacy level so that the epidemic curve can be flatten and hence it is possible for the country's health system to avoid being overwhelmed [12, 13].

Mathematical modelling in epidemic diseases has a long history, and many researchers adopted various types of models to investigate the dynamic behavior of the transmission of the disease [13]. Thanks to the advanced developments in computer technology in the modern era, efficient computer programs can be used to numerically simulate these mathematical models to test the level of efficacy of public health control measures, investigate the impact of vaccination and treatment programs, and obtain optimal resource allocation methods against outbreaks. Mathematical models following the compartmental structure, for instance, SIR (susceptible, infected, and recovered) or SEIR (susceptible, exposed, infected, and recovered), have been very popular among the researchers in mathematical epidemiology as they seem to be flexible in adjusting to describe a given disease dynamics.

A considerable amount of works that have adopted classical compartment models to instigate COVID-19 dynamic can be found. Most of them have used deterministic models, and various individual impact public health measures and other nonpharmaceutical interventions have been introduced in the parameter level, for instance, testing the efficacy of wearing masks to protect against the virus [14, 15].

In this study, we aim to adopt an SEIR (susceptible, exposed, infected, and recovered) type of a mathematical model to describe the COVID-19 dynamic in Sri Lanka, especially focusing on investigating the efficacy of aggregated control measures against the disease transmission and their timing of implementation to the community during the first few months of the outbreak. The model is further extended by addressing the heterogeneity of patients through the introduction of an intermediate class of patients who are likely to become critically ill from the disease and seek intensive care treatments [16]. Scenario-based control measures are developed, and they are introduced to the mathematical model. The numerical simulations are carried out to show how these measures are effective and also to predict the dynamic for a shorter period of time so that the health system can prepare accordingly.

## 2. Material and Methods

We apply a “susceptible-exposed-infected-recovered” (SEIR) framework to model the dynamic of the COVID-19 outbreak in Sri Lanka. We introduce two models basically; that is, the first model is an adaptation of a basic SEIR model using the traditional approach without considering the demography of patients. A new compartment is included to the model which represents the returnees to the country from abroad who are likely to be exposed to the virus overseas. However, in the second model, we introduce the new class of cases that includes the patients who may receive the intensive medical care due to the severity of the infection they undergo.

## 3. Mathematical Models

### 3.1. Model 1: SAEIR Model considering the Homogeneity of Patients

In this mathematical model, we assumed that all the clinically tested positive patients for COVID-19 virus are homogeneous with no impact of age, gender, and history of chronic diseases on the disease progression. Natural birth and death process was considered to be negligible, and those who recovered have developed complete immunity against the virus. In this simple model, the susceptible individual may become exposed to the novel coronavirus at a rate of *β*. After passing the time to show the symptoms of COVID-19 or time to identify clinically as positive to the virus*σ*, this exposed individual is designated as infected. As a result of treatments or due to the immunity, the patient can recover at a rate of *γ*; however, the patients whose condition is critical can end up losing their lives at a rate of *μ*. In the context of Sri Lanka, the island got the virus mainly from people who arrived from the overseas countries. Thus, we introduce a new compartment *A* representing the class of people who arrived to the island from overseas. Further, we let *λ* be the rate of new arrivals through the airport, *k*_1_ be the net rate of returned individuals who are cleared as negative to the virus and become again susceptible, and *k*_2_ be the net rate of returned individuals who are tested and clinically identified as infected. After 17 March 2020, the government introduced the mandatory quarantine requirement of all the overseas returned travelers immediately after their arrival to the country. Thus, we assume their ability to transmit the virus to the community is negligible. This dynamic can now be represented as follows given by the schematic diagram in Figure 1.

The mathematical model having the compartmental structure can be described as follows:

(1) $$\begin{array}{c} \frac{dS}{dt}=-\beta SI+k_{1}A,\\ \frac{dA}{dt}=\lambda -k_{1}A-k_{2}A,\\ \frac{dE}{dt}=\beta SI-\sigma E,\\ \frac{dI}{dt}=\sigma E+k_{2}A-\gamma I-\mu I,\\ \frac{dR}{dt}=\gamma I, \end{array}$$

with nonnegative initial conditions (*S*_0_, *E*_0_, *A*_0_, *I*_0_, *R*_0_).

### 3.2. Deriving the Basic Reproduction Number (*R*_0_)

The disease-free equilibrium (DFE) is basically given by (*S*_0_, 0, 0, 0, 0). According to the model in system (1), there are two infected classes of humans (*E* and *I*). We use the next-generation matrix method to find the basic reproduction number (*R*_0_) described in [17]. We derive the gains to *E* and *I* classes, respectively, as *βSI* and *σE*; similarly, we derive the losses from *E* and *I* classes as *σE* and (*γ* + *μ*)*I*, respectively. Now, we define the two matrices *F* and *V* such that

(2) $$\begin{array}{c} F={\left[\begin{array}{cc} \frac{\partial }{\partial E}\beta SI & \frac{\partial }{\partial E}\sigma E\\ \frac{\partial }{\partial I}\beta SI & \frac{\partial }{\partial I}\sigma E \end{array}\right]}_{\text{DFE}}=\left[\begin{array}{cc} 0 & \sigma \\ \beta S_{0} & 0 \end{array}\right],\\ V={\left[\begin{array}{cc} \frac{\partial }{\partial E}\sigma E & \frac{\partial }{\partial E}\left(\gamma +\mu \right)I\\ \frac{\partial }{\partial I}\sigma E & \frac{\partial }{\partial I}\left(\gamma +\mu \right)I \end{array}\right]}_{\text{DFE}}=\left[\begin{array}{cc} \sigma & 0\\ 0 & \left(\gamma +\mu \right) \end{array}\right]. \end{array}$$

Now, *FV*^−1^ is the next-generation matrix and *R*_0_ = *ρ*(*FV*^−1^), where *ρ*is the spectral radius. Thus, for system (1), the basic reproductive number is derived as *R*_0_ = *S*_0_*β*/(*γ* + *μ*) [17, 18].

## 4. Simulation of Model 1

The numerical simulation of the conceptual models for COVID-19 transmission is carried out in MATLAB, and the outcomes are shown in Figure 2. It should be noted that a hypothetical value for the transmission probability *β* is used for the simulation and no control measures are included for the simulation. According to the simulation of model 1, the nearly 55 days after the first local patient is found, the curve attains its peak.

### 4.1. Model 2: *SAEI*_m_*I*_c_*R* Model considering the Heterogeneity of Patients (including the Class of Patients Who Will Require ICU Treatments)

In this mathematical model, we have assumed that the clinically tested positive patients for COVID-19 are not homogeneous and took into consideration their age, gender, and history of chronic diseases that worsen severity and lead to ICU treatment [16]. The new group of patients *I*_c_ is added to the model representing the severe cases of COVID-19. These severe patients are absorbed by the available ICU beds until they reach the capacity.

According to this model, the recovery can happen in two ways. First, the patients in the *I*_m_ class may show mild symptoms of COVID-19 and eventually, all of them recover fully. Second, the condition may become severe based on the patients age, gender, lifestyle (smoking or alcohol addicted), and presence of chronic diseases. However, they recover due to the ICU treatment they receive while a small proportion die. While all other parameters are the same, the new parameters are introduced to the model such that *δ* is the rate at which a patient's level becomes critical. This should be in a measurable functional form with respect to several demographic variables. Further, *γ*_1_ is the recovery rate of patients who show mild symptoms while *γ*_2_ is the recovery rate of severely ill patients who are treated in ICUs where *γ*_1_ > *γ*_2_. In this model, the parameter *u* ∈ (0, 1) is the control parameter and it depends on multiple control and social distancing variables. It is further assumed that the patients in the ICU are isolated from the public and they are not responsible for the community transmission [13, 16]. The dynamic can now be represented according to the following schematic diagram (Figure 3).

The new model can now be stated as follows:

(3) $$\begin{array}{c} \frac{dS}{dt}=-\left(1-u\right)\beta {SI}_{\text{m}}+k_{1}A,\\ \frac{dA}{dt}=\lambda -k_{1}A-k_{2}A,\\ \frac{dE}{dt}=\left(1-u\right)\beta {SI}_{\text{m}}-\sigma E,\\ \frac{{dI}_{\text{m}}}{dt}=\sigma E+k_{2}A-\gamma_{1}I_{\text{m}}-\delta I_{\text{m}},\\ \frac{{dI}_{\text{c}}}{dt}=\delta I_{\text{m}}-\gamma_{2}I_{\text{c}}-\mu I_{\text{c}},\\ \frac{dR}{dt}=\gamma_{1}I_{\text{m}}+\gamma_{2}I_{\text{c}}. \end{array}$$

Following the same method described for system (1), the basic reproduction number for system (2) can be obtained as *R*_0_ = ((1 − *u*)*S*_0_*β*)/(*γ*_1_ + *δ*) assuming the critically ill patients are fully isolated and biologically, they are unable to transmit the virus anymore [16, 19].

### 4.2. Simulation of the *SAEI*_m_*I*_c_*R* Model (Model 2) with Critically Ill Patients

#### 4.2.1. Sensitivity of the Control Measures

The aim of this model is to assess the efficacy of control measures; however, the timing of control measures is not included in the simulation. We vary the control parameter *u* which addresses the combined impact of government social distancing control measures [20]. The outcome of this simulation is given in Figure 4. It can be seen that as the efficacy of the control measure increases, the epidemic curve is flattened and also, it is possible to delay the peak of the outbreak so that the national health system is able to treat patients without getting overwhelmed [16].

Figure 5 shows how it is possible to reduce the maximum of the curve representing the patients who show mild symptoms and the maximum of the curve representing critically ill patients for the given period of time. The figure clearly shows that the size of this peak reduces as the combined control parameter *u* is increased from 30% to 80%.

#### 4.2.2. Sensitivity of the Control of Overseas Exposed Cases

The government of Sri Lanka decided to minimize the rate of imported exposed cases to the island five days after the first local COVID-19 patient was identified. However, the authorities were flexible and allowed the arrival of Sri Lankan citizens from selected countries for further about three days and thereafter, the decision was made to shut down the international airport for all arrivals to the country. We analyze the effect of this decision from the model simulation though the parameter *λ*. We define this parameter as a step function in time such that

(4) $$\begin{array}{c} \lambda =\left\{\begin{array}{c} 0.041505,\;t<5,\\ 0.006105,\;5\leq t<8,\\ 0.000003,\;t\geq 8, \end{array}\right. \end{array}$$

where *t* is the number of days after the first Sri Lankan case of COVID-19 was identified by the health authorities in the country [12]. The outcome of this simulation is given in Figure 6.

Figure 7 shows how the peaks of the infected curve can be reduced with respect to the decision made to stop international arrivals who can be exposed to the virus.

#### 4.2.3. Sensitivity of the Timing of Implementing Combined Control Measures

It is very critical to introduce social distancing control measures in correct points in time to minimize the burden of COVID-19 [18]. Most of the EU countries have found to have misjudged the scheduling of these measures, and they have ended up with collapsing their health system causing a significantly large number of COVID-19 deaths. For this simulation, we vary the time in days from the date the first local case was identified until the government decided to impose drastic social distancing control measures (80% efficacy). It is assumed that until this date, the authorities were very flexible and they are at a mild level of restrictions (20% efficacy) [16, 18].  Figure 8 shows how the dynamic is changed with respective to this time parameter denoted by Tr.  Figure 9 demonstrates its sensitivity to both mild and critical case peaks.

According to Figure 8, it is very clear that this threshold value in time is very critical to minimize the burden to this highly contagious COVID-19. It suggests that if the government had introduced 80% social distancing control measures within 5 days of the first local case was identified, we may have prevented the steeper growth of cases and reduced the size of the peak significantly. The model also demonstrates that if we wait nearly for 30 days to impose control measures, then we are likely to experience a large peak of cases.  Figure 9 illustrates the relationship between time to introduce measures and the peak of cases showing how rapidly it grows with each delay.

## 5. Discussion and Conclusion

The simulations hypothetically show that if policymakers toughen the control measures, they can delay the peak and thereby flatten the curve. This will enable the health care system in the country to cope with both mild and severely ill patients of COVID-19. However, these recommendations are provided based on this early study with the proviso that the epidemic in the country is less than a month old and it is too early to make firm medium-term predictions [21].

It is important and relevant to identify and evaluate the current efficacy level of average aggregated combined social distancing measure as a percentage in Sri Lanka. The outbreak predication may be based on these values. With hindsight, one could argue that drastic control measures at the very beginning may have prevented the disease from getting established and spreading, e.g., banning all inward travels immediately after the first patient was detected. Of course, this was considered impractical with the available knowledge at the time. Similarly, severe restriction of movement of people with strict enforcement of curfews may eradicate the disease. However, practically, people have to be allowed to buy essential provisions and curfews have to be lifted for a few houses. As a result, the efficacy level of restricted mobility is never going to be perfect and continuous with respect to time.

Considering the complexity and uncertainty, we have mathematically modelled the control parameter with respect to various social distancing factors. We have also predicted the outbreak with respect to identified determinants of various combinations of social distancing and public health measures introduced in different ranges [20]. In addition, the results show that the timing of control measures taken into action is critical; that is, if the government decided to minimize the human movements early in the outbreak, then the epidemic curve could be flatten and the cases could be kept within the bounds that the health system can effectively manage.

It is also vital to check the timing (schedule) of control measures in effect during the active outbreak period through the simulation as we have learnt that if the country passes a certain point, then it has been unable to control the transmission regardless of how serious measures are being taken later. Finally, the literature from China found that only 20% of patients have developed the disease to critical stage requiring ICU care while others had less severe or mild or asymptomatic conditions of the disease. Therefore, in the public health perspective, it would be helpful to come up with a way to model and predict the patients who may become critically ill and seek ICU treatments considering multiple demographic factors.

## Figures and Tables

**Figure 1:** Schematic of model 1.

**Figure 2:** Simulation of model 1 without any control measures. The parameter values used for the simulation are *β* = 0.7, *γ* = 0.24, *μ* = 0.001, *σ* = 1/4, *λ* = 0.000205, *k*_1_ = 0.6, and *k*_2_ = 0.4 [13].

**Figure 3:** Schematic of model 2.

**Figure 4:** The simulation of model 2 considering the varying levels of the control parameter *u*. The rest of the parameter values used for the simulation are *β* = 0.7, *γ*_1_ = 0.24, *γ*_2_ = 0.05, *μ* = 0.02, *σ* = 1/4, *δ* = 0.025/3, *λ* = 0.000205, *k*_1_ = 0.6, and *k*_2_ = 0.4 [13, 19].

**Figure 5:** The change in the peak of mild cases and critical cases with respect to the combined control parameter *u*.

**Figure 6:** The simulation of model 2 considering the varying levels of the control parameter *u* and the time effect of the decision to shut down the airport. The rest of the parameter values used for the simulation are *β* = 0.7, *γ*_1_ = 0.24, *γ*_2_ = 0.05, *μ* = 0.02, *σ* = 1/4, *δ* = 0.025/3, *λ* = 0.000205, *k*_1_ = 0.6, and *k*_2_ = 0.4 [13, 16, 18, 19].

**Figure 7:** The change in the peak of mild cases and critical cases with respect to the combined control parameter *u* and the decision made to stop overseas exposed cases.

**Figure 8:** The simulation of model 2 considering the varying threshold time to impose strong social distancing control measures.

**Figure 9:** The change in the peak of mild cases and critical cases with respect to the threshold time to impose strong social distancing control measures.

## Data Availability

The data used to support the findings of this study are included within the manuscript.

## References

[1] Drosten C., Günther S., Preiser W. (2003). Identification of a novel coronavirus in patients with severe acute respiratory syndrome. *The New England Journal of Medicine*.

[2] Zaki A. M., van Boheemen S., Bestebroer T. M., Osterhaus A. D. M. E., Fouchier R. A. M. (2012). Isolation of a novel coronavirus from a man with pneumonia in Saudi Arabia. *The New England Journal of Medicine*.

[3] Hu B., Zeng L. P., Yang X. L. (2017). Discovery of a rich gene pool of bat SARS-related coronaviruses provides new insights into the origin of SARS coronavirus. *PLoS Pathogens*.

[4] Wang H., Li X., Li T. (2020). The genetic sequence, origin, and diagnosis of SARS-CoV-2. *Nature Public Emergency collection, European Journal of Clinical Microbiology & Infectious Diseases*.

[5] Fang Y., Nie Y., Penny M. (2020). Transmission dynamics of the COVID-19 outbreak and effectiveness of government interventions: a data-driven analysis. *Journal of Medical Virology*.

[6] Wu J. T., Leung K., Leung G. M. (2020). Nowcasting and forecasting the potential domestic and international spread of the 2019-nCoV outbreak originating in Wuhan, China: a modelling study. http://www.thelancet.

[7] Li Q., Guan X., Wu P. (2020). Early transmission dynamics in Wuhan, China, of novel coronavirus-infected pneumonia. *New England Journal of Medicine*.

[8] Nishiura H., Kobayashi T., Miyama T. (2020). Estimation of the asymptomatic ratio of novel coronavirus infections (COVID-19). *International Journal of Infectious Diseases*.

[9] Yang L., Yan L.-M., Wan L. (2020). Viral dynamics in mild and severe cases of COVID-19. *The Lancet Infectious Diseases*.

[10] Zhao S., Lin Q., Ran J. (2020). Preliminary estimation of the basic reproduction number of novel coronavirus (2019-nCoV) in China, from 2019 to 2020: a data-driven analysis in the early phase of the outbreak. *International Journal of Infectious Diseases*.

[11] Wu J. T., Leung K., Bushman M. (2020). Estimating clinical severity of COVID-19 from the transmission dynamics in Wuhan, China. *Nature Medicine*.

[12] http://www.epid.gov.lk/web/index.php?option=com_content&view=article&id=225&Itemid=518&lang=en

[13] Lin Q., Zhao S., Gao D. (2020). A conceptual model for the coronavirus disease 2019 (COVID-19) outbreak in Wuhan, China with individual reaction and governmental action. *International Journal of Infectious Diseases*.

[14] Eikenberry S. E., Mancuso M., Iboi E. (2020). To mask or not to mask: modeling the potential for face mask use by the general public to curtail the COVID-19 pandemic. *Infectious Disease Modelling*.

[15] Ngonghala C. N., Iboi E., Eikenberry S. (2020). Mathematical assessment of the impact of non-pharmaceutical interventions on curtailing the 2019 novel coronavirus. *Mathematical Biosciences*.

[16] Ferguson N. M., Laydon D., Nedjati-Gilani G. (2020). *Impact of non-pharmaceutical interventions (NPIs) to reduce COVID-19 mortality and healthcare demand*.

[17] Driessche P. V. D. (2017). Reproduction numbers of infectious disease models. *Advancing Research Evolving Science*.

[18] Hellewell J., Abbott S., Gimma A. (2020). Feasibility of controlling COVID-19 outbreaks by isolation of cases and contacts. *The Lancet Global Health*.

[19] Boldog P., Tekeli T., Vizi Z., Dénes A., Bartha F. A., Röst G. (2020). Risk assessment of novel coronavirus COVID-19 outbreaks outside China. *Journal of Clinical Medicine*.

[20] Prem K., Liu Y., Russell T. W. (2020). The effect of control strategies to reduce social mixing on outcomes of the COVID-19 epidemic in Wuhan, China: a modelling study. *The Lancet Public Health*.

[21] Kucharski A. J., Russell T. W., Diamond C. (2020). Early dynamics of transmission and control of COVID-19:a mathematical modelling study. *The Lancet Infectious Diseases*.

